# Incidence and Predictors of Pressure Ulcers among Adult Patients in Intensive Care Units at Arba Minch and Jinka Hospitals, Southern Ethiopia

**DOI:** 10.1155/2023/9361075

**Published:** 2023-04-15

**Authors:** Lankamo Ena Digesa, Ararso Baru, Alemayehu Shanko, Mekidim Kassa, Zeleke Aschalew, Fikre Moga, Bereket Beyene, Tegegn Mulatu

**Affiliations:** ^1^School of Nursing, College of Medicine and Health Sciences, Arba Minch University, Ethiopia; ^2^School of Medicine, College of Medicine and Health Sciences, Arba Minch University, Ethiopia; ^3^School of Public Health, College of Medicine and Health Sciences, Arba Minch University, Ethiopia

## Abstract

**Introduction:**

The incidence of a pressure ulcer in intensive care units (ICU) is significantly higher than in noncritical care settings. The patients in the ICU are the most vulnerable group to disruption of the skin's integrity. Prior studies in Ethiopia failed to evaluate pressure ulcers in intensive care units and were limited to general wards. The purpose of this study was to identify the incidence and predictors of pressure ulcers in adult patients admitted to intensive care units in Southern Ethiopia.

**Methods:**

A single-arm prospective open cohort of 216 patients was used to determine the presence of a pressure ulcer in the intensive care units from June 2021 to April 2022. A consecutive sampling was used until the sample size was reached. The data were collected using a structured questionnaire and analyzed using Stata 14. A cumulative incidence of a pressure ulcer was computed. The life table was used to estimate the cumulative survival. A multivariable Cox proportional hazard regression was used to identify independent predictors of a pressure ulcer. An adjusted hazard ratio with a 95% CI was used to measure the degree of association; a *P* value ≤ 0.05 was considered significant.

**Results:**

Twenty-five patients developed a pressure ulcer (PU), making a cumulative incidence of 11.57%. Out of 25 incident cases of pressure ulcers, four-fifths (80%) of the study patients developed PU within 6 days of their admission to the ICUs. The incidence rate was 32.98 PU per 1000 person-days of ICU stay. Pressure ulcers were most commonly found on the sacrum, followed by the shoulder. Among the incident cases, 52% were stage 2 ulcers. The presence of friction or shearing forces, as well as being 40 years of age or older, was independently associated with pressure ulcers.

**Conclusion:**

The overall cumulative incidence of the pressure ulcer was lower than that in other studies but occurred at a faster rate. Age (40 years of age or older) and the presence of friction or shearing forces were the main predictors of pressure ulcers in the intensive care units. Therefore, nurses working in ICUs should continually anticipate the risk of a pressure ulcer. Moreover, special attention should be given to patients of advanced ages. Furthermore, monitoring the installation of a mattress, keeping bed linens unwrinkled, and keeping patients in a proper position on a bed to prevent or reduce friction or shearing forces are very crucial in the prevention of pressure ulcers.

## 1. Introduction

A pressure ulcer is a type of skin damage that is limited to a specific area [1]. The soft tissue is damaged when it is pressed between bony prominence areas and an external surface [2]. A pressure ulcer is a major concern in today's intensive care units (ICUs) [3, 4]. Furthermore, a pressure ulcer is a main problem in nursing care, has a significant impact on the health care system, reduces the quality of life, exposes the patient to additional costs, complicates the patient's health condition, and is associated with a poor outcome in the ICU [2, 5–8].

A study showed that the cumulative incidence of pressure ulcers in adult ICU patients ranged from 10% to 25.9% [3]. Nevertheless, according to another systematic review, up to 49% of critically ill patients develop pressure ulcers [9]. According to numerous study reports from European and Brazilian intensive care units, the incidence ranged from 8.1% to 29.6% [10–14]. However, Asian intensive care units reported a higher cumulative incidence, ranging from 31.4% to 39.3% [15–17]. On the other hand, the lower cumulative incidence reported from African intensive care units ranges from 15% to 26.8% [18, 19].

Patients in intensive care units are more disadvantaged and vulnerable to the skin integrity disruption than non-ICU patients [6, 9, 11, 20, 21]. Several studies found that the incidence of pressure ulcers in intensive care patients was significantly higher than in non-ICU settings [6, 9, 13, 15, 18, 20–24]. According to a 2018 systematic review and meta-analysis in adult intensive care patients, the incidence of a pressure ulcer in adult ICU and non-ICU patients was 16.9%–23.8% and 12%–18%, respectively [3].

Previous studies showed that advanced age, smoking, an increased hospital stay, limited mobility, malnutrition, comorbidities, using vasoactive medications, pressure ulcer preventive devices, and friction or shearing forces were found to be the predictors of a pressure ulcer in the ICU [9, 11, 17, 25–28].

Identifying predictors associated with pressure ulcers in intensive care units is the foundation for preventing pressure ulcers. Previous research found differences in the incidence of pressure ulcers in intensive care units across countries. Moreover, prior studies in Ethiopia [26, 27, 29–32] failed to evaluate pressure ulcers in the intensive care units. Thus, there was insufficient data on pressure ulcers in Ethiopian intensive care units to adequately describe the problem. As a result, the purpose of this study was to identify the incidence and predictors of pressure ulcers in adult patients admitted to intensive care units in Southern Ethiopia.

## 2. Materials and Methods

### 2.1. Study Areas and Context

The study was carried out at the Arba Minch and Jinka Hospitals in Southern Ethiopia. Arba Minch and Jinka are administrative towns of the Gamo and South Omo Zones, respectively. Arba Minch and Jinka are 454 and 691 kilometers south of Addis Ababa, respectively. Based on 2017 population projections, the Gamo Zone projected a figure of 1,595,057 [33], while the South Omo Zone projected a figure of 722,955. The hospitals were selected because they were the only general hospitals that had intensive care units with wide catchment areas serving the zones and surrounding zones with a radius of 100 to 150 km. The number of admissions to the intensive care units varies. However, the estimated monthly admission for both intensive care units ranges from 32 to 35.

### 2.2. Study Period

The data were collected from June 2021 to April 2022.

### 2.3. Study Design

A single-arm prospective open cohort was used.

### 2.4. Source Population

Patients attending the intensive care units in the study hospitals.

### 2.5. Study Population

All the patients who were admitted to the intensive care units fulfilled the inclusion criteria.

### 2.6. Eligibility Criteria

#### 2.6.1. Inclusion Criteria

15 years of age or older.

#### 2.6.2. Exclusion Criteria

The patients who had pressure ulcers on admission were excluded from the study. Patients with dermatologic conditions also did not participate in this study, as these make the diagnosis difficult.

### 2.7. Sample Size Determination and Sampling Technique

The sample size was calculated using a previous study from Rwanda [19] with the following assumptions: the incidence of pressure ulcers in the ICU (15%), a 95% confidence level, and a margin of error of 5%. With a 10% nonresponse rate, the calculated sample size was 216. A consecutive sampling was used until the sample size was reached.

### 2.8. Operational Definitions

*Pressure ulcer*: having a stage one to four ulcer or an unstageable ulcer in one or more bony prominence areas during the follow-up period [2, 34].

*Censored*: a study participant who had a nonpressure ulcer outcome during the follow-up period (discharged without a pressure ulcer, death, transfer, or referral).

*Incidence of the pressure ulcer*: how many patients developed pressure ulcers during the follow-up period?

*Friction or shearing force*: the presence of wrinkles in bed linen or mattresses, tiny particles irritating the skin on the patient's linen, or the patient sliding down in a bed, when examining the patient [2].

*Comorbidities*: the condition of having two or more diseases simultaneously.

*Vasoactive active medication (phenylephrine, norepinephrine, epinephrine, vasopressin, dopamine, dobutamine, and milrinone)*: one or more medications that cause vasoconstriction and/or decreased perfusion [2, 35, 36].

*Pressure-relieving device*: any device that cushions pressure at bony prominence areas (pillows, cotton rings, water- or air-filled gloves, etc.) or the use of oil or moisturizing cream [8, 27].

### 2.9. Study Variables

#### 2.9.1. Dependent Variable

Pressure ulcer.

#### 2.9.2. Independent Variables

The independent variables are as follows: age, sex, body mass index, diagnosis at admission, comorbidities, smoking, length of stay at a hospital, position changing, friction or shearing forces, incontinence, vasoactive medications, and a pressure-relieving device.

### 2.10. Data Collection Instrument

A structured English-language questionnaire was used to collect the data. The data collection instrument was prepared based on previous studies [8, 13, 22, 25–27, 29, 30, 37] and the Waterlow scale, which is a widely used pressure ulcer risk assessment scale [1, 2]. The Waterlow scale is more suitable for pressure ulcer risk prediction in an intensive care unit than other scales [38]. The Waterlow scale has seven domains to assess the risk of a pressure ulcer: age and sex, BMI, continence, mobility, skin appearance in risk areas, nutrition, and special risks, with a higher score indicating a higher risk of developing a pressure ulcer. The face and content validity of the data collection instrument were thoroughly reviewed by subject area experts with specialties in critical care and emergency medicine in addition to the authors. The data collection instrument comprises baseline predictors, prognostic and therapeutic predictors, and the Waterlow pressure ulcer assessment scale. According to the European Pressure Ulcer Advisory Panel grading scale [34], pressure ulcers are classified into four stages and are unstageable. The data were collected by four senior BSc nurses from wards other than intensive care units and supervised by two MSc health professional supervisors. Daily until the discharge, referral, or death and the end of data collection, a comprehensive skin assessment from the head to toe was performed. The baseline data were gathered at the start of the study. For the updated care plan, the patient's records were reviewed, and document analysis was performed.

### 2.11. Data Quality Assurance

Before the actual study began, a pretest was conducted on 5% of the sample size at Ottona Teaching and Referral Hospital, Wolaita Sodo Town. After the pretest, modifications were made to the layout and wording of the questionnaire. Supervisors and data collectors received training on the KoboToolbox and data collection instrument. The trained supervisors checked the completeness of each questionnaire and the accuracy of the data during data collection.

### 2.12. Data Processing and Analysis

The data were collected by the KoboToolbox and analyzed by Stata version 14. A patient's status with a pressure ulcer was dichotomized as “pressure ulcer” or “censored” based on the patient's last contact. A descriptive analysis was done, including a measure of central tendency and frequency distribution for the categorical data. A cumulative incidence and an incidence rate were calculated. The life table was used to estimate the cumulative survival. A log-rank test was used to compare survival between different categories of independent variables. A bivariable Cox proportional hazard model was used to select the variables for multivariable analysis. A multivariable Cox proportional hazard model was fitted with the variables having a *P* value < 0.2 in the bivariate analysis. The predictors, which were the candidates for multivariable analysis, were checked for multicollinearity by the variance inflation factor (1.048 to 1.498) and correlation matrix before the statistical adjustment in the multivariable Cox regression model. The goodness of fit of the model was assessed using the Schoenfeld residuals, and a global test was used (0.7596). An adjusted hazard ratio with a 95% CI was used to measure the degree of the association, and statistical significance was declared at a *P* value ≤ 0.05.

### 2.13. Ethical Clearance

The ethical clearance was obtained from Arba Minch University, College of Medicine and Health Sciences, Institutional Research Ethics Review Board (IRB), with a reference number of IRB/1008/21. The letters of support were given to the concerned administrative bodies of the study hospitals. Permission to access intensive care units was received from the chief executive officer, medical director, and ICU coordinator. All ICU staff were informed about the study. The objective of the study was explained. Depending on the condition of the study participants, verbal informed consent was obtained. Consent was obtained from the study participant if he or she was conscious; if the participant was unconscious and sedated, consent was obtained from the surrogate (a relative or family member) if one was available or as per the study hospital's protocol for ICU administration. The name of the study participant was not written on the questionnaire. The study participant was coded anonymously, and confidentiality of information was maintained.

## 3. Results

### 3.1. Baseline Predictors of a Pressure Ulcer

This study included 216 adult patients who did not have pressure ulcers at the time of admission. The participants ranged in age from 15 to 88 years old. The study patients' median and interquartile range (IQR) ages were 30 and 19.5 years, respectively. Approximately half (52.31%) of the study participants were male. According to the Waterlow score, 100 (46.3%) of the study patients were at risk of developing a pressure ulcer at the time of admission to the intensive care units, as shown in Table 1.

### 3.2. Prognostic and Therapeutic Variables of a Pressure Ulcer

Two-thirds (67.59%) of study participants had no pressure-relieving devices at their bony prominence areas, as shown in Table 2.

### 3.3. The Incidence of Pressure Ulcers in the Intensive Care Units

Out of 216 ICU patients who were followed prospectively, 25 developed pressure ulcers, yielding a cumulative incidence of 11.57%. Others were referred, died, or were transferred to wards or discharged from the ICUs after they improved. The patients were followed for a minimum of one day and a maximum of eighteen days. Out of 25 incident cases of pressure ulcers, four-fifths (80%) of the study patients developed PU within 6 days of their admission to the ICUs. The cohort contributed to a total of 758 person-days of follow-up. Pressure ulcers occurred at a rate of 32.98 per 1000 person-days of ICU stay. The cumulative probability of survival at the end of the first, sixth, and eighteenth days was 0.9948, 0.7385, and 0.208, respectively, as shown in Table 3.

Nearly the same proportion of the incident cases was stage two and stage one, 13 (52%) and 12 (48%), respectively. As shown in Table 4, the sacrum (84%) was the most commonly affected site, followed by the shoulder (60%).

### 3.4. Comparison of Survival Probability among Categories of Covariates

A log-rank test was used to assess the existence of significant differences in survival probability between the various categories of variables. Accordingly, the age, Waterlow score, positioning, friction or shearing forces, and pressure-relieving devices were found to be significant at *P* < 0.05, as shown in Table 5.

### 3.5. The Predictors of a Pressure Ulcer in the Intensive Care Units

The study participants who were 40 years of age or older had a threefold higher risk of developing a pressure ulcer than their counterparts. Moreover, having friction or shearing forces was associated with a 4-fold higher hazard of a pressure ulcer than not having friction or shearing forces, as shown in Table 6.

## 4. Discussion

According to the findings of this study, the cumulative incidence of a pressure ulcer was 11.57% (7.92%, 16.61%). The result was comparable to research findings from Rwanda [19], Poland [14], Spain [12], and the systematic review [3]. On the contrary, the outcome was lower than previous studies conducted in Cameroon [18], Lebanon [15], Saudi Arabia [17], Brazil [11, 13], Italy [39], and Canada [6]. The difference could be due to the smaller size of the studies in Brazil, Saudi Arabia, Lebanon, and Italy, which may overestimate the incidence. Furthermore, the differences may be attributed to nursing staff awareness and training, vigilant teamwork, and adherence to protocols for pressure ulcer prevention strategies. However, because the intensive care units in our study had limited bed numbers, patients may have been discharged too quickly, underestimating the incidence of pressure ulcers.

According to this study, the overall incidence rate of pressure ulcers was 32.98 per 1000 person-days of ICU stay. The finding was higher than the incidence rate reported by studies in Spain [12] and Italy [39]. This indicates that the incidence rate of pressure ulcers in this study was faster than that in the reported studies. This was confirmed by the fact that the majority (80%) of the study patients developed PU within a few days or six days of their admission to the intensive care units.

The result of this study revealed that the patients aged 40 years or older had a 3-fold (AHR: 2.73 (1.087–684)) higher risk of developing a pressure ulcer than their counterparts. The finding was consistent with studies from Saudi Arabia [17], Ethiopia [26, 27], Brazil [13], and ICU pressure ulcer reviews [2, 40]. According to a Brazilian study, however, age was not associated with a pressure ulcer [11]. This is justified by the fact that elderly people have lower subcutaneous fat, a thinner dermis, and poor sensory perception and are less likely to respond to tissue signals to shift positions [2].

The presence of friction or shearing forces increased the risk of a pressure ulcer by four times (AHR: 4.47 (1.54–12.94)) compared to the absence of friction or shearing forces. Ethiopian studies [29, 30], Brazilian studies [25], and an ICU review [2] all confirmed the finding. This is justified by the fact that critical patients are immobile with little or no response to stimuli, increasing the risk of friction and shearing forces [12].

According to the findings of this study, the sacrum was the most commonly affected site (84%). Previous studies from Rwanda [19], Saudi Arabia [22], and Italy [39] supported the finding. This could be because the vast majority of patients are positioned semi- or Fowler's supine with no pressure-relieving devices, resulting in increased pressure points on the sacrum [17].

## 5. Limitations of the Study

The study's intensive care units had limited bed numbers, which may result in a rapid discharge rate, which may affect the incidence of a pressure ulcer. Since we used consecutive sampling, this might affect the generalizability of the findings. The variables were only recorded while the patients were in the intensive care units; no data were obtained after they were discharged. Moreover, the study did not look at the effect of clinical or medical devices on pressure ulcers. Furthermore, using the Cox hazard regression on a small number of outcome events or pressure ulcers may affect the findings' generalizability. However, survival analysis provides a better understanding of a pressure ulcer.

## 6. Conclusion

The overall cumulative incidence of the pressure ulcer was lower than that in other studies but occurred at a faster rate. Among the incident cases of pressure ulcers, four-fifths (80%) of the study patients developed pressure ulcers within 6 days of their admission to the ICUs. In the intensive care units, advanced age and the presence of friction or shearing forces were found to be predictors of pressure ulcers. Therefore, when caring for critically ill patients, nurses in intensive care units must constantly anticipate the risk of developing a pressure ulcer. Special consideration should be given to patients of advanced ages. Furthermore, a correct mattress installation, keeping bed linens unwrinkled and smooth, avoiding small particles irritating the skin, and keeping patients in a proper position on a bed are very important for the prevention or reduction of friction or shearing forces. Future research should focus on tertiary or comprehensive intensive care units.

## Figures and Tables

**Table 1:** Baseline variables of the pressure ulcer among adult patients admitted to intensive care units at Arba Minch and Jinka Hospitals, Southern Ethiopia, 2021/2022.

Variable	Category	Survival status		
		Censored (%)	PU (%)	Total (%)
Sex	Male	99 (45.83)	14 (6.48)	113 (52.31)
	Female	92 (42.59)	11 (5.1)	103 (47.69)
Age	<40 years	143 (66.20)	10 (4.63)	153 (70.83)
	≥40 years	48 (22.22)	15 (6.94)	63 (29.17)
Body mass index (BMI)	Normal weight	172 (79.63)	21 (9.72)	193 (89.35)
	Overweight	19 (8.8)	4 (1.85)	23 (10.65)
Level of consciousness at admission (in GCS)	≥13	115 (53.24)	17 (7.87)	132 (61.11)
	≤12	76 (35.19)	8 (3.70)	84 (38.89)
Waterlow score within 6 hours of admission (PU risk calculator)	<10	112 (51.85)	4 (1.85)	116 (53.70)
	≥10	79 (36.57)	21 (9.72)	100 (46.30)
Smoking	No	185 (85.65)	24 (11.11)	209 (96.76)
	Yes	6 (2.78)	1 (0.46)	7 (3.24)
Comorbidity	No	160 (74.07)	20 (9.26)	180 (83.33)
	Yes	31 (14.35)	5 (2.32)	36 (16.67)

The Waterlow score < 10 denotes less risk and ≥10 denotes at risk, high risk, and very high risk. GCS: Glasgow Coma Scale; PU: pressure ulcer; comorbidity: having two or more diseases simultaneously.

**Table 2:** Prognostic and therapeutic variables of the pressure ulcer among adult patients admitted to intensive care units at Arba Minch and Jinka Hospitals, Southern Ethiopia, 2021/22.

Variable	Category	Survival status		
		Censored (%)	PU (%)	Total (%)
Frequent positioning	No	26 (12.04)	9 (4.16)	35 (16.2)
	Yes	165 (73.39)	16 (7.41)	181 (83.8)
Friction or shearing forces	No	185 (85.65)	7 (3.24)	192 (88.89)
	Yes	6 (2.78)	18 (8.33)	24 (11.11)
Incontinence (fecal or/and urine)	No	136 (62.96)	19 (8.8)	155 (71.76)
	Yes	55 (25.46)	6 (2.78)	61 (28.24)
Pressure-relieving device (at bony prominence areas)	No	138 (63.89)	8 (3.70)	146 (67.59)
	Yes	53 (24.54)	17 (7.87)	70 (32.41)
Vasoactive medications	No	176 (81.86)	25 (11.57)	201 (93.06)
	Yes	15 (6.94)	0 (0)	15 (6.94)

PU: pressure ulcer.

**Table 3:** The life table for survival among adult patients admitted to intensive care units at Arba Minch and Jinka Hospitals, Southern Ethiopia, 2021/22.

Time in day	Number of patients at the beginning	Lost	Number of pressure ulcers	Survival	95% CI
1	216	50	1	0.9948	0.9634, 0.9993
2	165	52	8	0.9375	0.8830, 0.9671
3	105	25	1	0.9274	0.8681, 0.9606
4	79	19	4	0.8740	0.7906, 0.9257
5	56	19	3	0.8176	0.7107, 0.8881
6	34	6	3	0.7385	0.6014, 0.8347
7	25	12	0	0.7385	0.6014, 0.8347
9	13	1	2	0.6203	0.4175, 0.7702
10	10	1	1	0.5550	0.3369, 0.7272
11	8	1	0	0.5550	0.3369, 0.7272
12	7	1	0	0.5550	0.3369, 0.7272
14	6	1	0	0.5550	0.3369, 0.7272
15	5	1	0	0.5550	0.3369, 0.7272
16	4	0	1	0.4163	0.1518, 0.6654
18	3	2	1	0.2081	0.0152, 0.5552

**Table 4:** Locations of the pressure ulcer among adult patients admitted to intensive care units at Arba Minch and Jinka Hospitals, Southern Ethiopia, 2021/22.

Location of pressure ulcer	Frequency	Percentage	Cumulative
Sacrum	9	36	36
Shoulder and sacrum	8	32	68
Shoulder, sacrum, and elbow	3	12	80
Shoulder, sacrum, elbow, and heel	1	4	84
Shoulder	1	4	88
Elbow and shoulder	2	8	96
Elbow	1	4	100
Total	25	100	

**Table 5:** A log-rank test of the study variables among adult patients admitted to intensive care units at Arba Minch and Jinka Hospitals, Southern Ethiopia, 2021/22.

Variables	Chi 2 (*X*^2^)	*Pr* > chi 2
Sex	0.74	0.3885
Age	11.55	0.0007
BMI	1.35	0.2450
Admission GCS	1.23	0.2672
Waterlow score within 6 hours of admission	4.98	0.0257
Smoking	0.00	0.9545
Comorbidity	0.76	0.3846
Frequent positioning	7.41	0.0065
Friction or shearing forces	47.41	0.0000
Incontinence (fecal or/and urine)	2.54	0.1110
Pressure-relieving device (at bony prominence areas)	10.27	0.0014
Vasoactive medications	2.90	0.0886

**Table 6:** Multivariable analysis among adult patients admitted to intensive care units at Arba Minch and Jinka Hospitals, Southern Ethiopia, 2021/22.

Variable	Category	Survival status		CHR (95% CI)	AHR (95% CI)	*P* value
		Censored (%)	PU (%)			
Age	<40 years	143 (66.20)	10 (4.63)	1.0		
	≥40 years	48 (22.22)	15 (6.94)	3.6 (1.6-8.02)	2.73 (1.08-6.84)	0.032
Waterlow score within 6 hours of admission (PU risk calculator)	<10	112 (51.85)	4 (1.85)	1.0		
	≥10	79 (36.57)	21 (9.72)	3.2 (1.06-9.66)	2.76 (0.82-9.29)	0.102
Frequent positioning	No	26 (12.04)	9 (4.16)	2.9 (1.28-6.77)	0.56 (0.199)	0.261
	Yes	165 (73.39)	16 (7.41)	1.0		
Friction or shearing forces	No	185 (85.65)	7 (3.24)	1.0		
	Yes	6 (2.78)	18 (8.33)	11.8 (4.85-28.58)	4.47 (1.54-12.9)	0.006
Incontinence (fecal or/and urine)	No	136 (62.96)	19 (8.8)	1.0		
	Yes	55 (25.46)	6 (2.78)	0.48 (0.188-1.23)	0.48 (0.18-1.28)	0.143
Pressure-relieving devices	No	138 (63.89)	8 (3.70)	3.56 (1.53-8.30)	2.77 (0.99-7.76)	0.052
	Yes	53 (24.54)	17 (7.87)	1.0		

The Waterlow score < 10 denotes less risk and ≥10 denotes at risk, high risk, and very high risk. AHR: adjusted hazard ratio; CHR: crude hazard ratio; PU: pressure ulcer.

## Data Availability

The datasets used to support the findings of this study are available from the corresponding author upon request.
